The article "Associations Between Gross Motor Coordination and Executive Functions: Considering the Sex Difference in Chinese Middle-Aged School Children" was published in 2022. Journal: Front Psychol.

# Associations Between Gross Motor Coordination and Executive Functions: Considering the Sex Difference in Chinese Middle-Aged School Children

**DOI:** 10.3389/fpsyg.2022.875256

**Published:** 2022-06-22

**Authors:** Shijie Liu, Si-Tong Chen, Yujun Cai

**Affiliations:** ^1^School of Physical Education and Sport Training, Shanghai University of Sport, Shanghai, China; ^2^Institute for Health & Sport, Victoria University, Melbourne, VIC, Australia

**Keywords:** gross motor coordination, executive functions, children, working memory, inhibition function

## Abstract

Considering that motor and cognitive processes are intertwined and inhibit or help each other throughout life and that primary school age is one of the most critical stages of children's cognitive and motor development, this study aimed to investigate the relationship between executive functions and gross motor skills in Chinese children aged 9–10 years, as well as gender differences. The flanker task, the 1-back task, the more-odd shifting task, and the test of gross motor coordination (Körperkoordinationtest für Kinder) were used to collect data on executive functions and gross motor coordination. The results were as follows. First, there was a weak association between gross motor coordination and the inhibition reaction time in the congruent test and the reaction time of working memory (*r* = −0.181 to −0.233), but no association was found between gross motor coordination and cognitive flexibility. Second, a weak-to-moderate correlation was presented between the move sideways test and the inhibition reaction time in the congruent test and the reaction time in the refreshing test of the working memory (*r* = −0.211 to −0.330). Finally, gender influenced on the relationship between gross motor coordination and the reaction time of both inhibition (β_Gender_ = −0.153, *p* < 0.05) and working memory (β_Gender_ = −0.345, *p* < 0.01). To conclude, our results suggest that children with better motor coordination skills require less reaction time, especially girls, and this association was more substantial than in boys. The finding supports the current assertion that there are commonalities between gross motor coordination and cognitive control by showing the relationship between gross motor coordination and complex cognitive processes (executive function) in preadolescent children.

## Introduction

Gross motor coordination (GMC) represents the involvement of large body muscles in balance, limb, and trunk movements (Chaves et al., 2016). It is a complex trait that integrates internal neurological and neuromotor processes (Keogh and Sugden, 1985), and its manifold expression is generally explained in terms of additive genetic effects, as well as their interaction with environmental factors (Chaves et al., 2016). Well-developed GMC goes hand-in-hand with higher levels of complex movement and sport-specific skills, which are essential for developing higher levels of cognitive function (Irene and Vander-Fels, 2015). Executive functions (EFs) are cognitive processes that influence actions, ideas, and emotions from top to bottom (Zelazo and Carlson, 2012) and include attentional or cognitive flexibility, working memory, and inhibitory control, which enable individuals to plan, organize, and solve problems, as well as to manage their impulses (Best and Miller, 2010). It is also known as complex cognitive functions (i.e., higher-level cognitive processes that control and regulate complex cognitive processes) (Su et al., 2021). Low GMC levels were shown to be related to complex cognitive functions and language development in children and adolescents (Houwen et al., 2016). Additionally, more and more scholars encourage starting from the “exercise benefits intelligence” theory hypothesis, which states that motor and cognitive skills are intertwined and inhibit or help each other throughout life (Piaget and Cook, 1952; Payne and Labban, 2017). Therefore, GMC is not only an important aspect of children's motor development but also of their cognitive growth.

The article "Associations Between Gross Motor Coordination and Executive Functions: Considering the Sex Difference in Chinese Middle-Aged School Children" was published in 2022. Journal: Front Psychol.

In recent years, the impact of exercise on children's EF has been the focus of international scholars. A growing body of research has explored the benefits of short-term (Chang et al., 2012; Vera and Emi, 2016), long-term (Ludyga et al., 2018; Liu et al., 2020), and a variety of traditional physical activities (Egger et al., 2018; Gu et al., 2021) on children's EF (Verburgh et al., 2014). Recently, within the preadolescent age range, several meta-analyses have shown that enhanced cognitive functioning as a result of physical activity is most obvious in EFs (Verburgh et al., 2014; Liu et al., 2020) and attention (Greeff et al., 2017).

Several underlying mechanisms might explain the effects of physical activity on EF. From a psychophysiological perspective, acute physical activity can cause an increase in neurotransmitters (e.g., epinephrine, dopamine, brain-derived neurotrophic factors), which are thought to enhance EF processes (Dishman et al., 2006; Roig et al., 2013). Additionally, relevant brain research has also verified the positive effect of physical activity on individual cognitive processes, which can improve EF and attention in adolescents. Physical activity promotes strong self-regulation ability and goal-oriented behavior, enabling adolescents to effectively plan, manage, and implement multiple tasks, and enhances their ability to adapt to the external environment (Vandenbroucke et al., 2018). These findings provide more scientific evidence for the role of exercise in complex and advanced cognitive development in children.

The article "Associations Between Gross Motor Coordination and Executive Functions: Considering the Sex Difference in Chinese Middle-Aged School Children" was published in 2022. Journal: Front Psychol.

For years, different views have been expressed about the relationship between GMC and EF in children and adolescents. Rigoli, Piek, Kane, and Oosterlan reported positive associations of motor coordination (MC) with working memory and inhibitory control in children aged 12–16 years and found that GMC and EF presented a linear association (beta = 0.29, *p* < 0.05) (Rigoli et al., 2012). Carlos, Luz, and Luis showed that 9–11-year-old children with high MC have better cognitive performance and found a moderate correlation between gross motor [Körperkoordinationtest für Kinder (KTK)] coordination and EF (CAS) (Carlos et al., 2014). However, Livesey et al. (2006) showed that gross motor skills (MABC) in children aged 5–6 years were only weakly related to response inhibition (Stroop and stop-signal task). Unfortunately, these studies did not consider the expected effects of MC on EF in linear regression. However, the current literature has indicated the relationship between motor skills (MOBAK-5) and working memory in children aged 10–12 years, and no relationship has been found in inhibition control and motor skills and in switching tests and any type of motor skills (Ludyga et al., 2019). In contrast, another recent study demonstrated that among the components of EFs (BRIEF), inhibition, working memory, planning/organizing, and organization had a significant relationship with gross motor skills (TGMD-2) in children aged 8–10 years, with success rates of 48, 39, 25, and 43%, respectively, and found locomotor and EF presented a linear association [beta = 0.56, *p* < 0.01; (Athirezaie et al., 2022)]. This laid the foundation for the research hypothesis to test the regression relationship between GMC and EF.

Findings from these previous studies on the relationship between EF and gross motor skills have not been unified. It is possible that the GMC assessment tools of these studies, including refined motor skills (MABC, TGMD), led to different results. Moreover, EF varies greatly in adjacent age groups of children, and there is a lack of research on the relationship between EF and GMC in children at certain ages. Therefore, the relationship between GMC and EF in children needs to be further explored, especially in the single age group of children aged 9–10 years. To the best of our knowledge, the relationship between GMC and EF in Chinese children has not been investigated. This may be related to the lack of development of assessment tools for GMC in Chinese children and adolescents. Therefore, we adopted the KTK, which is an overall dynamic coordination assessment for children and adolescents aged 5–14 years, which has been adopted by researchers worldwide (Vandorpe et al., 2011). Moreover, the accuracy and reaction time of the EF in this test are remarkable. Some studies have confirmed that MC has different correlations with reaction time and EF accuracy (Xu and Yan, 1999), but previous studies do not finely distinguish the behavioral data of EF. Therefore, it was necessary for this study to explore the potential relationship between EF accuracy, reaction time, and GMC based on previous studies. Furthermore, previous studies have shown that there is no gender difference in children's EF (Welsh et al., 1991), but other studies have found that white boys respond faster than white girls, black boys, and black girls when they complete the go/no-go task (Brocki and Bohlin, 2004). The GMC of different genders also has certain differences (Moreira et al., 2019), so it seems that the effects of gender on EF and GMC also need to be considered.

The article "Associations Between Gross Motor Coordination and Executive Functions: Considering the Sex Difference in Chinese Middle-Aged School Children" was published in 2022. Journal: Front Psychol.

Based on the above, our study has three objectives, namely, (1) to determine the GMC and EF of children aged 9–10 years in China; (2) explore the correlation between GMC and EF in children aged 9–10 years; and (3) study gender and body mass index (BMI) differences in the relationship of GMC and EF. Hopefully, our study can enrich the empirical research on the correlation between children's GMC and EF.

## Research Method

### Participants

As the forerunner of the integrated reform of physical education in China, Shanghai has a strong representation in China. Participants were recruited from two public primary schools in Shanghai by convenience sampling, L and N. It was found that the assessment standards of P.E. lessons from the two public schools in 2019 and 2020 were consistent with the overall standards of all schools in Shanghai, and there was no statistically significant difference between the two public schools mentioned above, which meant that the research samples reflected the overall situation of primary schools in Shanghai.

The research samples (*n*) included 364 healthy children aged 9–10 years (the percentage of girls: 46.1%) (average age: 9.55 ± 0.92 years). Data for another six children were excluded because of reported motor impairment (*n* = 2) or absence on test days (*n* = 4). The Gpower3.1 statistical software was utilized to analyze obtained data. The study first supposed effect size = 0.50, α = 0.05, and statistical test power = 0.90, then presented the minimum sample size as 290. Given the 20% inefficiency rate caused by MC and invalid measurement of EF, the final sample size was 364.

The article "Associations Between Gross Motor Coordination and Executive Functions: Considering the Sex Difference in Chinese Middle-Aged School Children" was published in 2022. Journal: Front Psychol.

Several points should be clarified. (1) All children participated in the study of their own accord, and only when parents provided written consent and children themselves verbally agreed to participate in this study. (2) All the children were sighted or obtained corrected visual acuity, and no neuromuscular disease was found. (3) The participants enjoyed normal development of intelligence without mental or learning disabilities as assessed by their teachers. (4) All procedures complied with the Declaration of Helsinki. (5) The study was authorized by the Institutional Review Board of the local Education Department (102772021RT072), which takes responsibility for evaluating the research conducted in schools.

### Research Tools and Procedures

#### Procedures

All participants were tested separately in quiet rooms at their respective institutions. From September to November 2020, 364 children aged 9–10 years were tested for GMC and EF. The testers consisted of 22 graduate students (education major, second-year graduate students) who familiarized themselves with children's motor skills, test procedures, and standard language by watching relevant test videos, and pre-tested 40 non-tested children. During the pretest, testers gave oral guidance and demonstrations as required. Finally, an experienced and well-trained experiment leader evaluated the testers' performances. The evaluation included three parts, namely, oral guidance, demonstration, and test procedures. Moreover, as the KTK tool is an outcome assessment tool, the assessment was conducted by three researchers. Two researchers separately conducted field tests. When there was disagreement between the two researchers, a third researcher evaluated the original video to reach a consensus.

Two stages were involved in the test, namely, (1) measurement of gross motion coordination from September to October 2020 and (2) measurements of EF were scheduled between 12:45 p.m. and 13:15 p.m. and took place in groups of 20 in a school classroom in November 2020.

#### Children's GMC (KTK Tool)

The KTK assessment tool of GMC was adopted in this study. Schilling, a German scholar, revised it for the second time in 2007 and reported that the KTK reliability coefficients of a single test ranged from 0.80 to 0.96; the coefficient of the total battery was 0.97 (Vandorpe et al., 2011). The reliabilities in this study (intraclass correlations) varied between 0.753 and 0.782 per dimension (Song, 2020), which was higher than the internal consistency pass line (0.7) set by Nunnally (Nunally, 1978; Hair et al., 1995; Wu, 2003), and retested reliability varied between 0.832 and 0.961. The KTK consists of four subtests lasting for 15–20 min for each participant. Details are presented as follows.

(1) Jumping sideways (JS). The jump side task consists of a field (60 × 100 cm) framed by sidelines and divided into two halves by a center line. Participants were required to complete as many sideways jumps as possible, with feet together, over a wooden slat (two trials, each for 15 s). A child's jump on one of the lines was not counted. Ultimately, we added up the number of jumps for both trials. Notably, these jumps were performed using two legs.
(2) Moving sideways (MS). Participants were required to move across the floor for 20 s using two wooden platforms (e.g., cross the first board, reach the second board, move the first board, and step on the second board), and participants had two opportunities. To ensure that children moved sideways, two 50-cm-long boundaries were added. Ultimately, we added up the number of jumps for both trials.
(3) Hopping for height (HH). Participants hopped on one leg over an increasing number of 5 cm foam blocks to a maximum of 12 blocks. Participants began hopping 1.5 m away from the foam blocks, hopped up to and over the foam block, and completed a further two hops for the trial to be deemed successful. Three trials were given for each height, with 3, 2, or 1 point(s) given for a successful performance during the first, second, or third trial, respectively.
(4) Walking backward (WB). In this task, children were instructed to walk backward along three balance beams with differences in width (3 m length; 5 cm height; 6, 4.5, and 3 cm widths). A maximum of 24 steps (8 per trial) was counted for each balance beam, which comprised a maximum of 72 steps (24 steps × 3 beams) for this test. The number of successful steps on each beam was calculated.

The article "Associations Between Gross Motor Coordination and Executive Functions: Considering the Sex Difference in Chinese Middle-Aged School Children" was published in 2022. Journal: Front Psychol.

The original score for overall MC was calculated by adding the original scores of the four subtests into a formula. Based on guidance for the latest edition of the KTK in 2007, the original score of overall MC was converted according to the reference [motor quotient (MQ)] of specific age and gender, hence obtaining the MQ (Hair et al., 1995; Wu, 2003; Vandorpe et al., 2011). Records with scores significantly deviating from the standard were verified, and tests missed by participants were conducted at another time.

#### Executive Function

Our study adopted the measurement tool of children's EF (validity > 0.85) developed by Chen Aiguo et al. in 2011 (Zhang et al., 2017). Participants were seated in front of a laptop (with 80 cm distance between participants) and completed computer-based versions of flexibility, working memory, and inhibitory control exercises, which were administered with the E-Prime software 1.1 (Psychology Software Tools, Pittsburgh, USA).

The flanker task was employed to assess inhibitory function, including congruent and incongruent trials. A congruent test consisted of a horizontal array with the same five letters, such as LLLLL or FFFFF, whereas an incongruent test consisted of a horizontal array of five letters with different middle letters, such as LLFLL or FFLFF. In inhibition tasks, participants were required to press F or L with their left or right index finger according to the middle letters that appeared in the trial. Pressing the wrong button or failing to react within the specified time was considered an incorrect reaction. Participants were asked to perform 12 pre-trials and then complete two modes with 48 trials. Each mode had an interval of 1 min. Tests, both congruent and incongruent, were conducted in a random order with equal probability in each group. The duration was about 6 min for two modes. A smaller score for reaction times or higher accuracy meant better inhibition ability.

The 1-back task was employed to assess working memory, which included a series of rapidly changing letters (B, D, L, Y, O) presented at the center of the computer screen for 2 s with an interval of 3 s. Participants carefully observed each letter and determined whether it was the same letter as the one that had appeared before the two trials. If so, they pressed the “F” key; if not, they pressed the “L” key. Identical and different letters each accounted for 50%. Pressing the wrong button or failing to react within 1.5 s was considered an incorrect reaction. The trial consisted of two stages every 25 times. A shorter reaction time indicated better working memory, and higher accuracy meant refreshing ability.

The more-odd-shifting task was employed to assess cognitive flexibility. A number appeared in the center of the computer screen every 2 s, and the participants were asked to make judgments of the presented numbers (1–9). The task consisted of three sections, namely, (a) “big or small” – a black number was presented on the screen. If the number presented was smaller than 5, they pressed the “F” key; otherwise, they pressed the “L” key. (b) “Odd or even” – a green number was presented on the screen. If the number presented was even, they pressed the “L” key; otherwise, they pressed the “F” key. (c) This section contained type A and B tests. Participants were asked to press the “F” or “L” key to indicate whether the black numbers were greater than 5 and whether the green numbers were odd or even. The trial was divided into six sections with the sequence of “abccba.” Segments A and B did not need to be switched, each presenting 16 times. Segment C was switched 32 times, including 16 switch processes. A pretest was conducted 8 times for segments A and B and 16 times for segment C the first time. The test results measured the difference in reaction time between the switching condition (the average of segment C) and the non-switching condition (the average of segments A and B). Smaller differences and higher accuracy signified better cognitive flexibility.

The article "Associations Between Gross Motor Coordination and Executive Functions: Considering the Sex Difference in Chinese Middle-Aged School Children" was published in 2022. Journal: Front Psychol.

#### BMI Test

The BMI test requires subjects to use the Ogilvy Health electronic body mass and height meter (Sengkang Jiaye HK6800 children's version; the unit is accurate to 0.01 kg and 0.01 cm) in the state of underwear and bare feet, and the obtained data are passed through BMI = kg/m^2^ to calculate the BMI value for each child.

### Statistical Analysis

The *t*-test was performed on the subjects' gross motor scores and EF to test for gender differences. Using the Pearson product-moment correlation coefficient and two-tailed *p* < 0.05 was considered statistically significant for a difference. Correlations were calculated between subjects' GMC and inhibition, working memory, and cognitive flexibility. Finally, by controlling for gender variables, linear regression analysis was performed with gross motor scores as independent variables, EF total scores and inhibition, working memory, and cognitive flexibility as dependent variables.

Before analysis, the normal distribution, linearity, and homogeneity of variance were verified by an independent-samples *t*-test using a histogram, P-P plot, and scatter plot (Tabachnick and Fidell, 2014), and the test level was *p* = 0.05. According to Cohen's classification, the correlation (*r*) was divided into weak (*r* = 0.10), moderate (*r* = 0.30), and high (*r* = 0.50), whereas effect size (*R*^2^) was classified as weak effect (1–8%), moderate effect (9–24%), and strong effect (≥25%).

## Results

### Descriptive Statistics of Children's GMC and EF

The descriptive statistics of GMC and EF with gender differences are shown in Table 1. Before analysis, we used the histogram to perform the normality test, the histogram tends to be normally distributed, and the distribution curve is centered. The average of motor quotient for GMC was 84.56 (12.95). In terms of gender-based differences in GMC, boys outperformed girls in jumping sideways and hopping for height (*p* < 0.05). In walking backward and moving sideways, girls were better than boys, and there were also statistical differences (*p* < 0.05).

**Table 1:** Descriptive statistics of gross motor coordination and executive function of children aged 9–10 years.

**Variables**	**Boys (*n* = 196)**	**Girls (*n* = 168)**	**Total (*n* = 364)**	**Gender difference (*T*)**	**Gender difference (*p)***
BMI	18.98 (3.63)	16.91 (2.82)	17.98 (3.42)	−1.38	0.003^2)^
Gross motor coordination					
MQ	86.45 (15.56)	82.17 (12.97)	84.56 (12.95)	−2.94	0.027^1)^
WB	38.25 (5.43)	44.95 (9.64)	39.96 (7.87)	−4.41	0.016^1)^
HH	35.58 (4.56)	29.17 (2.97)	30.21 (2.49)	−0.340	0.030^1)^
JS	45.54 (13.78)	38.94 (13.20)	41.66 (13.55)	−0.146	0.046^1)^
MS	11.47 (3.05)	15.81 (3.26)	13.40 (3.28)	3.09	0.005^2)^
GMC	127.18 (34.95)	121.71 (17.79)	123.93 (32.08)	−1.46	0.145
Executive function					
***Inhibition***					
Reaction time of incongruent test	611.18 (95.28)	622.44 (86.05)	616.38 (91.19)	1.07	0.234
Reaction time of congruent test	630.28 (146.25)	609.08 (96.43)	620.49 ± 126.02	−3.78	0.000^2)^
Accuracy of incongruent test	0.83 (0.16)	0.81 (0.14)	0.82 (0.16)	−1.61	0.109
Accuracy of congruent test	0.84 (0.15)	0.88 (0.09)	0.86 (0.12)	1.42	0.156
***Working memory***					
Reaction Time of Refreshing Test	926.89 (159.03)	864.32 (160.21)	889.35 (178.91)	−4.17	0.010^1)^
Accuracy of Refreshing Test	0.75 (0.21)	0.88 (0.11)	0.77 (0.21)	2.57	0.005^2)^
***Cognitive flexibility***					
Reaction time of big–small/Odd–even test	829.89 (191.74)	807.01 (155.14)	819.33 (175.93)	−1.24	0.220
Reaction time of switching test	976.15 (137.28)	1231.54 (298.17)	1113.67 (269.59)	10.21	0.000^2)^
Accuracy of big–small/ odd–even test	0.52 (0.15)	0.73 (0.19)	0.77 (0.17)	2.72	0.047^1)^
Accuracy of switching test	0.55 (0.17)	0.61 (0.29)	0.57 (0.18)	2.45	0.015^1)^

*1) p < 0.05; 2) p < 0.01. MQ, motor quotient; WB, walking backward; HH, hopping for height; JS, jumping sideways; MS, moving sideways; GMC, gross motor coordination*.

The article "Associations Between Gross Motor Coordination and Executive Functions: Considering the Sex Difference in Chinese Middle-Aged School Children" was published in 2022. Journal: Front Psychol.

In terms of the EF, in the inhibition task, boys surpassed girls in reaction time in the congruent/incongruent tests and accuracy rate in the incongruent test, while girls outperformed in the reaction time in the congruent test and accuracy rate in the congruent test. Among them, statistical significance was found in the reaction time in the congruent tests (*p* < 0.05). In the refreshing test, the 1-back reaction time and accuracy of girls were better than those of boys with respective statistical significance (*p* < 0.01). As for cognitive flexibility, girls surpassed boys in accuracy in the switching and big-small/odd-even tests, both with statistical significance (*p* < 0.05).

### Correlation Between GMC and EFs

By drawing a scatter plot, it is intuitively judged that there is a linear relationship between the two, and by drawing a standardized residual scatter plot and a histogram and P-P plot with a standard curve, we believe that the residual variance is a homogeneous and approximately normal distribution. Correlation analysis (Table 2) showed a significantly weak correlation between MQ and inhibition reaction time and working memory reaction time (*r* = −0.181, *p* < 0.01; *r* = −0.232,*p* < 0.01). However, there was no significant correlation between the MQ and the accuracy of inhibition and working memory as well as cognitive flexibility (*p* > 0.05). In terms of inhibiting task response time, there was a statistically significant weak correlation between WB, MS, and congruent test response time for the total sample (*r* = −0.168 to−0.221, *p* < 0.01), while WB, MS, and MQ were statistically different and weak correlated with incongruent test response time for girls (*r* = −0.148 to −0.182, *p* < 0.05). In terms of accuracy, the JS enjoyed a significantly weak correlation with accuracy in the incongruent test (*r* = 0.136, *p* < 0.05), and the MS of girls had a remarkably weak correlation with accuracy in the incongruent test (*r* = 0.129, *p* < 0.05). In working memory, the MS of the whole sample was significantly and moderately correlated with the reaction time (*r* = −0.330, *p* < 0.01). Girls' WB was significantly different and weakly correlated with reaction time (*r* = −0.215, *p* < 0.01), and accuracy was statistically different and weakly correlated (*r* = 0.134, *p* < 0.05). There was a significant weak correlation between MS and working memory accuracy of girls (*r* = 0.181, *p* < 0.01). In addition, there was a statistically different and weak correlation between WB and accuracy in the girls' cognitive flexibility (*r* = 0.183, *p* < 0.05) and a statistically different and weak correlation between JS and cognitive flexibility reaction time in the girls (*r* = −0.148, *p* < 0.05).

The article "Associations Between Gross Motor Coordination and Executive Functions: Considering the Sex Difference in Chinese Middle-Aged School Children" was published in 2022. Journal: Front Psychol.

**Table 2:** Correlation between gross motor coordination and executive functions of children aged 9–10 years.

**Test**	**Gender**	**Inhibition**				**Cognitive flexibility**				**Working memory**	
		**Reaction time of**	**Reaction time of**	**Accuracy of**	**Accuracy of**	**Reaction time of**	**Reaction time of**	**Accuracy of**	**Accuracy of**	**Reaction time**	**Accuracy of**
		**incongruent**	**congruent**	**incongruent**	**congruent**	**big–small/**	**switching**	**big–small/**	**switching**	**of refreshing**	**refreshing**
		**test**	**test**	**test**	**test**	**odd–even test**	**test**	**odd–even test**	**test**	**test**	**test**
WB	Boys	−0.124	−0.159^1)^	0.078	0.12	0.036	−0.132	−0.068	−0.042	−0.026	−0.016
	Girls	−0.153^1)^	−0.185^2)^	0.006	0.038	−0.077	−0.096	0.079	0.183^1)^	−0.215^2)^	0.134^1)^
	Total	−0.113	−0.168^1)^	0.017	0.099	−0.039	−0.103	0.050	0.068	−0.108	0.036
HH	Boys	0.024	−0.074	0.058	0.112	−0.02	−0.068	−0.047	−0.062	−0.070	0.097
	Girls	−0.069	−0.009	−0.023	−0.007	0.016	−0.068	−0.102	0.054	−0.036	0.026
	Total	−0.013	−0.056	0.003	0.077	−0.013	−0.134	−0.076	0.029	−0.038	0.087
JS	Boys	−0.006	−0.049	0.108	0.059	−0.045	−0.084	−0.114	−0.126	−0.012	−0.025
	Girls	−0.034	−0.166^1)^	0.147^1)^	0.072	−0.073	−0.148^1)^	−0.085	−0.009	−0.134	0.033
	Total	−0.016	−0.09	0.136^1)^	0.064	−0.057	−0.094	−0.108	−0.066	−0.05	0.004
MS	Boys	−0.106	−0.181^1)^	0.051	0.09	0.007	−0.064	0.009	0.098	−0.271^2)^	0.047
	Girls	−0.182^1)^	−0.252^2)^	0.062	0.129^1)^	−0.05	−0.118	−0.044	−0.058	−0.354^2)^	0.181^2)^
	Total	−0.133	−0.211^2)^	0.038	0.115	−0.031	−0.099	0.043	0.067	−0.330^2)^	0.088
MQ	Boys	−0.105	−0.155^1)^	0.118	0.068	0.050	−0.011	−0.126	0.075	−0.186^2)^	0.033
	Girls	−0.148^1)^	−0.195^2)^	0.078	0.121	0.020	−0.080	0.102	0.030	−0.288^2)^	0.063
	Total	−0.116	−0.181^2)^	0.105	0.082	0.041	−0.055	−0.098	0.054	−0.233^2)^	0.045

*1) p < 0.05; (2) p < 0.01. MQ, motor quotient; WB, walking backward; HH, hopping for height; JS, jumping sideways; MS, moving sideways*.

The article "Associations Between Gross Motor Coordination and Executive Functions: Considering the Sex Difference in Chinese Middle-Aged School Children" was published in 2022. Journal: Front Psychol.

In summary, MQ and MS in children aged 9–10 years, there was a weak-to-moderate correlation with inhibition of control consistency reaction time, and reaction time of working memory. To further explore the effect of gross movement on inhibitory control and working memory, we took the reaction time in the congruent test of inhibitory function and the reaction time in the refreshing test of working memory as dependent variables (Table 3), multiple linear regression analysis was performed with gender and BMI as independent variables, MQ, or MS.

**Table 3:** Regression analysis of the correlation between gross motor coordination and executive functions of children aged 9–10 years.

**Task**	**Dependent variable**	**Variable**	***B***	**Standard error**	**β**	***t***	***p***	**VIF**	***R***	***R*** **^2^**	** $R_{\text{adj}}^{2}$ **	***F***
Inhibition	Reaction time of congruent test	MS	−0.558	0.379	−0.281	2.731	0.010^1)^	1.043	0.211	0.045	0.042	*F*_(3, 361)_ = 12.541, *p < * 0.05*
		Gender	−1.494	0.120	−0.153	2.115	0.024^1)^	2.096				
		BMI	0.020	0.683	0.021	0.055	0.178	2.053				
											*D*–*W* value	2.190
	Reaction time of congruent test	MQ	−0.893	0.463	−0.258	1.877	0.044^1)^	1.215	0.186	0.035	0.030	*F*_(3, 361)_ = 9.013, *p <* 0.05*
		Gender	−0.782	0.095	−0.187	1.561	0.155	1.808				
		BMI	−0.588	0.014	−0.069	1.120	0.178	2.348				
											*D*–*W* value	2.032
Working memory	Reaction time of refreshing test	MS	−0.872	0.520	−0.330	4.569	0.001^2)^	1.466	0.331	0.109	0.106	*F*_(3, 361)_ = 25.923, *p <* 0.01**
		Gender	0.521	0.866	−0.345	5.544	0.000^2)^	2.224				
		BMI	−0.216	0.480	−0.097	2.160	0.016^1)^	1.528				
											*D*–*W* value	1.789
	Reaction time of refreshing test	MQ	−0.427	0.647	−0.233^2)^	4.123	0.001^2)^	1.938	0.225	0.051	0.049	*F*_(3, 361)_ = 19.427, *p <* 0.01**
		Gender	−0.253	0.476	−0.201^2)^	1.943	0.020^1)^	2.175				
		BMI	−0.031	0.637	−0.081	0.055	0.297	1.250				
											*D*–*W* value	2.251

*(1) p < 0.05; (2) p < 0.01*.

The article "Associations Between Gross Motor Coordination and Executive Functions: Considering the Sex Difference in Chinese Middle-Aged School Children" was published in 2022. Journal: Front Psychol.

The MS had a weak and predictive effect on the reaction time in the congruent test (${\text{R}}_{\text{adj}}^{2}$ = 0.042, *p* < 0.05) of inhibitory control. Specifically, for each unit change in the MS, the reaction time in the congruent test changed by −0.281 standard deviation. The MQ had a weak and predictive effect on reaction time in the congruent test (${\text{R}}_{\text{adj}}^{2}$ = 0.030, *p* < 0.05). Specifically, for every unit change in the MQ, reaction time in the congruent test changed by −0.258 standard deviations. Furthermore, gender had a significant influence on the reaction time in the congruent test of inhibitory control (β = −0.153, *p* < 0.05). The MS had a moderate and predictive effect on the reaction time in the refreshing test of working memory (${\text{R}}_{\text{adj}}^{2}$ = 0.106, *p* < 0.01), that is, for every unit change in the MS, the reaction time in the refreshing test changed by −0.330 standard deviations. The MS had a stronger predictive effect on the reaction time in the working memory refresh test. In addition, the MQ had a weak and predictive effect on the reaction time in the refreshing test of working memory (${\text{R}}_{\text{adj}}^{2}$ = 0.049, *p* < 0.01), that is, for every unit change in the MQ, the reaction time in the refreshing test changed by −0.233 standard deviations. Moreover, gender and BMI explained 10.6% of the variation in reaction time in the refreshing test (*F*_(3, 361)_ = 25.923, *p* < 0.01), gender, and BMI (β_Gender_ = −0.345, *p* < 0.01; β_BMI_ = −0.097, *p* < 0.05) became the best variables to negatively predict the reaction time in the refreshing test.

## Discussion

The first goal of this study was to analyze the GMC and EF of children aged 9–10 years in China. According to descriptive statistics, the MQ of Chinese children aged 9–10 years [83.56 (12.95)] was lower than that of Australian children [90.60 (16.50)] and Belgian children [96.40 (13.40)] (Bardid et al., 2015), indicating that Chinese children have weaker GMC ability. The reason for this may be that Chinese children completed the KTK test more carefully, performed the test tasks too seriously, paid more attention to the completion of the test, and ignored the continuity of the skills (e.g., with the addition of two 50 cm long boundaries, children will pay more careful attention to these constraints).

The article "Associations Between Gross Motor Coordination and Executive Functions: Considering the Sex Difference in Chinese Middle-Aged School Children" was published in 2022. Journal: Front Psychol.

The scores for EF were similar to the statistics in the published studies on EF in Chinese children (Chen et al., 2015) because children's EF remains stable around the age of 10. This result was also supported by neuropsychological research (James, 1996). The result demonstrated that girls outperformed boys in the inhibition reaction time in the congruent test, reaction time and accuracy of working memory, accuracy in the big-small/odd-even tests and cognitive flexibility, while boys surpassed girls in the switching test. A possible explanation is that the subtests of inhibition and working memory tasks focused on simple reaction time, which is shorter in girls after the age of 9 than in boys (Li and Luo, 2012). Thus, girls between the ages of 9 and 10 performed better than boys in inhibition and refreshing tasks. On the contrary, the subtests of switching were dominated by the choice reaction time. Because of gender differences in reaction types based on different characteristics, boys generally have faster choice reaction times (Li and Luo, 2012), while girls may prefer to make cautious decisions, which also leads to higher accuracy.

The second goal of this study was to analyze the relationship between GMC and EF. In working memory, we found moderate associations between reaction time in the refreshing test and the MC (−0.33), and weak associations between reaction time in the refreshing test and the MQ (−0.23). Furthermore, in inhibition, we found weak associations between reaction time in the congruent test and the MC (−0.21) and MQ (−0.18). These results were weaker than the results reported by Davis et al. (2012) and Rigoli et al. (2012). Both studies used older children and standardized quantitative and qualitative measures for motor proficiency. It is worth emphasizing that Carlos et al. (2014) used standard cognitive assessment tools, and Ludyga et al. (2019) and our study used EF assessment tools, which are more focused on EF. Ludyga et al. (2019) evaluated children aged 10–12 years in Switzerland and found an association of (−0.31) between motor skills (MOBAK-5) and working memory.

Notably, differences in the measures used to assess EF and gross motor skills are common (e.g., MOBAK-5 aims to evaluate the quality of movement, which is process-oriented compared with the KTK, while MABC selects children with severe motor difficulties), which may account for the heterogeneity of results because of differences between product (e.g., KTK) and process-oriented (e.g., MOBAK-5) results. Additionally, there are many types of EF assessment tools. In this study, we focused on cognitive ability, and a recent study has targeted EF assessments (e.g., flanker task, go/no-go). Furthermore, we found that children with high quantitative MQ scores performed better in working memory tests. Some studies have also linked working memory performance to aerobic fitness rather than to motor competences (Raine et al., 2013; Marchetti et al., 2015). As fitness was not assessed in this study, it remains unclear whether this variable mediated the correlation between gross motor skills and working memory updating.

The article "Associations Between Gross Motor Coordination and Executive Functions: Considering the Sex Difference in Chinese Middle-Aged School Children" was published in 2022. Journal: Front Psychol.

After controlling for variables such as gender and BMI through regression analysis, it was found that the MS and MQ contributed 10.6 and 4.9%, respectively, to the reaction time in the refreshing test. The MS and MQ contributed 4.2 and 3.0%, respectively, to the inhibition reaction time in the congruent test. This indicated that compared with the WB, HH, and JS, the MS had a better predictive effect on EF. This may be related to the action characteristics of the MS, which emphasized cooperation of upper and lower limbs space orientation and balance. Moreover, the sensitivity of the individual may also be improved through good body posture adjustment, and the lower limbs, trunk, and upper limbs form an efficient and coordinated dynamic chain that promotes rapid changes in movement and direction. Therefore, when children completed the MS, they needed to map the given password and the actions they needed to perform, and according to the password change, new schemas were extracted to which they must respond accurately and quickly, which challenges their working memory and inhibition. In addition, the WB had a certain weak correlation with the reaction time in the congruent test of the inhibition. This was because when children performed the WB tasks, they could pay enough attention to the balance beam, which reflected the inhibition of the response. However, the HH belonged to the dimension of whole-body coordination. Although single-leg hopping required coordination between swinging and supporting the legs, since it was a one-time jump, it did not require high sustained attention. Completing the JS required a focus on strength and endurance. Although this skill involved physical coordination, children use it frequently in daily life, and for them, the task is relatively simple and therefore not significant. This may be related to what we found earlier, that the internal consistency of the KTK assessment tool for Chinese children was not high, and that there were differences in the measurement focus of these four items.

Coincidentally, in a recent study that included the KTK assessment tool and EF, Maurer (2019) pointed out that the performance of simple and difficult GMC tasks had differential effects with EF (Maurer, 2019). Given the non-association between the easy gross motor tasks (JS, HH) and EFs, we assume that the required GMC movements were not completely automated. Children in this age group have probably reached a point of skill development at which the EFs are no longer substantially required to perform the tasks (Carlson et al., 2013). Therefore, the EFs were likely to be minimally involved during the performance of the easy gross motor tasks (JS, HH), leading to their weak and non-significant association with EFs. The reason is that subtests such as the HH and JS are simple and are often used in P.E. classes, so the participants' high proficiency in these MC tasks leads to the weakening of the automatic reaction of EF. Therefore, gross motor skills must constantly change the context of the task. Only in the context of dynamic movement do individuals need inhibitory responses (Alesi et al., 2016).

The article "Associations Between Gross Motor Coordination and Executive Functions: Considering the Sex Difference in Chinese Middle-Aged School Children" was published in 2022. Journal: Front Psychol.

The mechanisms underlying the association between gross motor skills and EF are still a matter of an ongoing debate (Irene and Vander-Fels, 2015). Current literature has shown that children with high motor competences are more effective in guiding the preparation of complex MC structures (involving working memory operations) than those with low motor competences (Ludyga et al., 2018). In addition, previous studies have found a specific relationship between visuospatial memory and certain aspects of MC (Piek et al., 2008; Rigoli et al., 2012). It has been speculated that the MC of early gross motor skills is related to the development of later working memory abilities, and it has been speculated that these specific associations may be partly determined by a common cerebellar mechanism. In addition, previous studies have also offered explanations from the perspective of neural mechanisms; that is, the participation of neural pre-activation mechanisms is high, and motor skills with complex background environments can not only promote children's physiological arousal but also cause cognitive activation to a greater extent (Diamond, 2000). The ability to pre-activate neural networks related to cognition is reflected in the cognitive requirements of gross motor skills themselves. When gross motor tasks are difficult, novel, unmastered or practiced, varied rather than fixed, they must be focused rather than automated and require quick reflexes and responses so attention will be specifically activated, which can promote increased activity in the cerebellum and prefrontal regions.

No correlation existed between GMC and cognitive flexibility, but it does not mean that people can ignore the positive impact of GMC on cognitive flexibility. No correlation may be related to differences in the underlying neural processes of inhibition, working memory, and cognitive flexibility. Cognitive flexibility is a complex task, which requires participants to switch between operations and mental sets when performing complex tasks in addition to the inherent inhibition requirements, motor skills with higher complexity require a higher correlation between MC and cognitive flexibility (Cui et al., 2019). Cognitive flexibility has a longer development process than other EFs, and improvements in cognitive flexibility throughout childhood are delayed as was shown in other studies; 13-year-old children still have not reached the level of adults (Davidson et al., 2006). To date, similar to the results of this research, the studies mentioned above have reported either no correlation between these variables (Rigoli et al., 2012; Ludyga et al., 2019) or a weak correlation between cognitive flexibility and gross motor skills (Roebers and Kauer, 2009).

The article "Associations Between Gross Motor Coordination and Executive Functions: Considering the Sex Difference in Chinese Middle-Aged School Children" was published in 2022. Journal: Front Psychol.

Regarding the third goal of our study, the results indicated that gender exerts influence on the relationship between GMC and the reaction times of both inhibition and working memory. In the evaluation of EF, girls were better than boys in inhibition (reaction time in the congruent test) and working memory (reaction time in the refreshing test, accuracy in the refreshing test). This may be related to the gender differences in individual cognitive ability and brain development. The overall development of boys is later than that of girls. The gender differences in the cognitive development of 9-year-old children may stem from the development of individual physiological maturity and brain structure. In addition, the development of gross motor skills for 9–10 years old showed gender differences. Boys developed better in strength and physical skills, while girls developed better in physical coordination skills. Some methodological issues limited the interpretation of the present results. The present findings were based on a cross-sectional investigation, so causality could not be inferred.

In general, many factors cause differences between MC and EF. There remain flaws in this study, namely, (1) participants only included children aged 9–10 years in primary school. Differences in study stage, age, mental conditions, and socioeconomic backgrounds may have had an impact on the correlation of MC and EF, which deserves further research. (2) This study only considered the simple transmission mechanism of GMC and EF. In fact, there may be mediating effects and moderating effects of multiple variables concerning people's mental processes, so future research should include more mediators, including self-efficacy and self-regulation ability, to reflect the complex transmission process between GMC and EF. (3) As cross-sectional research, this study could not provide further information on the directional relationship between motor and cognitive areas. In the future, longitudinal studies on related topics should be conducted to provide more empirical evidence for the benefits of exercise for children's cognitive development.

The article "Associations Between Gross Motor Coordination and Executive Functions: Considering the Sex Difference in Chinese Middle-Aged School Children" was published in 2022. Journal: Front Psychol.

## Conclusion

By investigating the primary relationship between the GMC and EF of children aged 9–10 years in China, compared with cognitive flexibility and inhibitory control, GMC had a better-than-expected effect on working memory.

We found that children with better MC skills require less reaction time of working memory, especially girls, and this association was more substantial than in boys. MS was the most effective for EFs among the GMC. It is hoped that this study will demonstrate the benefit of improving gross motor skills in promoting the EF of children aged 9–10 years and provide a reference for relevant departments to formulate sound strategies for encouraging physical exercise for children and adolescents.

## Data Availability Statement

The original contributions presented in the study are included in the article/supplementary material, further inquiries can be directed to the corresponding author/s.

## Ethics Statement

The studies involving human participants were reviewed and approved by the Ethics Committee of the Shanghai University of Sport. Written informed consent to participate in this study was provided by the participants' legal guardian/next of kin.

## Author Contributions

SL, S-TC, and YC contributed to the conception and design of the study. SL and S-TC organized the database and performed the statistical analysis. S-TC and YC contributed to manuscript revision, read, and approved the submitted version. All authors contributed to the article and approved the submitted version.

## Funding

This study was supported by the 2020 Shanghai Educational Science Research Project (The Second Batch), Research on the Teaching Model of Higher Education Goal-Oriented Sports Skills: Taking Shanghai as an Example, project approval number: C2-2020029; and the Shanghai Key Lab of Human Performance (Shanghai University of Sport) (No. 11DZ2261100); and the 2021 Shanghai Local Institutions Capacity Building Project-Research on Key Technologies of Science and Technology to Assist Shanghai Competitive Gymnasts' Athletic Performance Enhancement (21010503700).

## Conflict of Interest

The authors declare that the research was conducted in the absence of any commercial or financial relationships that could be construed as a potential conflict of interest.

The article "Associations Between Gross Motor Coordination and Executive Functions: Considering the Sex Difference in Chinese Middle-Aged School Children" was published in 2022. Journal: Front Psychol.

## Publisher's Note

All claims expressed in this article are solely those of the authors and do not necessarily represent those of their affiliated organizations, or those of the publisher, the editors and the reviewers. Any product that may be evaluated in this article, or claim that may be made by its manufacturer, is not guaranteed or endorsed by the publisher.
